The article "Antidiarrheal Effect of 80% Methanol Extract and Fractions of Clerodendrum myricoides (Hochst.) Vatke (Lamiaceae) Leaf in Swiss Albino Mice" was published in 2021. Journal: Evid Based Complement Alternat Med.

# Antidiarrheal Effect of 80% Methanol Extract and Fractions of *Clerodendrum myricoides* (Hochst.) Vatke (Lamiaceae) Leaf in Swiss Albino Mice

**DOI:** 10.1155/2021/9369173

**Published:** 2021-10-19

**Authors:** Getaye Tessema Desta, Muluken Adela Alemu, Asegedech Tsegaw, Tafere Mulaw Belete, Baye Yrga Adugna

**Affiliations:** ^1^Department of Pharmacy, College of Medicine and Health Sciences, Debre Tabor University, Debre Tabor, Ethiopia; ^2^Department of Pharmacology, School of Pharmacy, College of Medicine and Health Sciences, University of Gondar, Gondar, Ethiopia; ^3^Department of Pharmacy, Amhara Regional Health Bureau, Bahir Dar, Ethiopia

## Abstract

**Background:**

Diarrhea is one of the tempting symptoms of diseases in the world. In Ethiopian traditional medicine practices, *Clerodendrum myricoides* is utilized for the treatment of diarrhea without scientific evidence.

**Objective:**

This study was aimed to evaluate the antidiarrheal activity of 80% methanol extract and fractions of the leaf of *Clerodendrum myricoides* in mice.

**Methods:**

The crude extract was prepared by maceration in 80% methanol and then fractionated using hexane, chloroform, and distilled water. Antidiarrheal activity was assessed by castor oil-induced diarrhea, enteropooling, and gastrointestinal motility models using onset of diarrhea, number and weight of feces, volume and weight of intestinal contents, and distance travelled by charcoal meal as main parameters. Negative controls received either distilled water or 2% Tween 80 (10 ml/kg), positive controls received 3 mg/kg loperamide or 1 mg/kg atropine, and the test groups received 100, 200, and 400 mg/kg doses of the extract.

**Results:**

The crude extract and chloroform fraction significantly prolonged the onset of diarrhea at 200 and 400 mg/kg and decreased the number of wet, total, and weight of fresh feces at all tested doses. Hexane fraction has a significant antidiarrheal effect on the onset, number, and weight of feces at 400 mg/kg. The crude extract and chloroform fraction at all tested doses, as well as aqueous fraction at 200 mg/kg and 100 mg/kg, produced significant reduction in volume and weight of intestinal contents. Additionally, hexane fraction showed significant reduction of volume and weight of the intestinal content at 400 mg/kg. In the gastrointestinal motility test model, both chloroform fraction and crude extract at all tested doses and aqueous fraction at 200 mg/kg and 400 mg/kg showed a significant antidiarrheal effect as compared to the negative control.

**Conclusion:**

The leaf of *Clerodendrum myricoides* showed antidiarrheal activity which supports the traditional use.

## 1. Introduction

Diarrhea is a global health problem affecting all regions and populations, particularly in low and middle income countries of sub-Saharan Africa and Asia from which very young and old aged are more vulnerable [1, 2].

The article "Antidiarrheal Effect of 80% Methanol Extract and Fractions of Clerodendrum myricoides (Hochst.) Vatke (Lamiaceae) Leaf in Swiss Albino Mice" was published in 2021. Journal: Evid Based Complement Alternat Med.

Globally in 2019, diarrhea is the 8^th^ leading cause of death among all ages, which is responsible for 1.6 million deaths and the second cause of death among children younger than 5 years and accounts for 760,000 children deaths annually [3]. The overall mortality rate is 22.4 deaths per 100,000 yearly. The highest rate of diarrhea mortality among children younger than 5 years occurred in Chad, Central African Republic, and Niger. In the same year, diarrhea caused about 694,010 deaths among those aged 70 years and older [4]. According to 2018 systematic meta-analysis study the prevalence of diarrhea among children under five in Ethiopia was 22% [5].

Diarrhea is one of the most prominent diseases treated by traditional medicines [6]. *C. myricoides* (Misirich in Amharic and Maraasisaa in Oromo) is an open shrub that is 6- to 10-feet tall and 6-feet wide with 4-inch-long dark green glossy leaves which are arranged opposite. Flowers are bilaterally symmetrical [7]. In Ethiopia, *C. myricoides* is used for the treatment of different diseases including diarrhea. The leaf and root are used for treatment of diarrhea by using water as a vehicle [8–11]. The root of *C*. *myricoides* is utilized for the management of gonorrhea, typhoid, epilepsy, arthritis, tonsils, cough/cold, and rheumatism, and the leaf is used for treatment of diabetes in the people of Kenya [12, 13]. The root part is indicated for urinary retention, malaria, toothache, liver, and cancer [14, 15], the root bark for dry cough, and the fresh leaf for epilepsy and black leg [16].

A number of *in vitro* studies were conducted on different parts of *C. myricoides*. Extract from the leaf of *C. myricoides* showed antibacterial activity against *Streptococcus pyogenes*, *Staphylococcus aureus*, and *Pseudomonas aeruginosa* [17]. The acetone extract of the leaf showed antioxidant activity with 84% free radical scavenging activity [18]. Methanol extracts from the root also showed a significant antioxidant activity using the 1,1-diphenyl-2-picrylhydrazyl [19]. Stem extract had showed antileishmanial activity [20]. The methanol extract of the leaf produced antimalarial activity against *Plasmodium berghei* in infected mice with 82.50% suppression [21]. The ethanol extract of the leaf possessed anticonvulsant activity in mice [22].

The current drugs used for treating diarrhea are accompanied by many problems, including adverse effects, drug-drug interactions, and contraindications. They are associated with hypersensitivity, drug interactions, and side effects like constipation, respiratory depression, lethargy, excitement, and coma [23, 24]. Some of the drugs are not affordable for the poor. Due to these, search for cheaper, safe, and effective new antidiarrheal medication better than the present drugs is crucial.

The article "Antidiarrheal Effect of 80% Methanol Extract and Fractions of Clerodendrum myricoides (Hochst.) Vatke (Lamiaceae) Leaf in Swiss Albino Mice" was published in 2021. Journal: Evid Based Complement Alternat Med.

The phytochemical screening on the methanol and the chloroform extract of leaf showed the presence of glycosides, tannins, steroids, alkaloids, saponins, phenols, flavonoids, and terpenoids [25, 26]. People around the world including Ethiopia utilized medicinal plants for the management of diarrhea. *C. myricoides* is one of the medicinal plants used for the treatment of diarrhea in different parts of Ethiopia [8–11] without scientific evaluation and proof on its efficacy. In addition to the traditionally claimed antidiarrheal use, there were *in vitro* tests on antioxidant and anti-inflammatory activities [26, 27] as well as phytochemical screening tests [27]. The safety of the leaf was established. Dichloromethane and methanol leaf extracts produced antimutagenicity activity against *Salmonella typhimurium* TA98 and TA100 bacterial strains [28–30]. Absence of scientific validation on the antidiarrheal activity of the leaf in living systems and the aforementioned evidence abetted carrying out this experiment in animal models. Additionally, the finding of this research could contribute as an input in searching for new antidiarrheal agent that might solve problems associated with the current antidiarrheal drugs.

## 2. Materials and Methods

### 2.1. Drugs and Chemicals

The following drugs and chemicals were used during this study: distilled water (University of Gondar Teaching Specialized Hospital, Ethiopia), loperamide hydrochloride (Medochemie Ltd, Limassol Cyprus), castor oil (Amman Pharmaceutical Industries, Jordan), methanol (Blulux, India), chloroform (Carlo Erba Reagents, France), hexane (Pentokey Organy, India), activated charcoal (Acuro Organics Ltd, New Delhi), Tween 80 (Atlas Chemical Industries Inc, India), and atropine sulfate injection (0.1%) (JeilPharm. Co. Ltd., Korea), Mayer's and Dragendorff's reagents (May and Baker Ltd, Dagenham, England), ferric chloride (BDH Ltd, England), potassium ferrocyanide (BDH Ltd, England), ammonia (Merck Millipore, India), acetic anhydride (Techno Pharmchem, India), lead acetate test (Fisher Scientific, UK), sulfuric acid (Farm Italia Carlo Erba, Italy).

### 2.2. Plant Material

The leaves of *C. myricoides* were collected from Teda around Gondar city, northwest Ethiopia, in December, 2019. The plant specimen was identified and authenticated by Dr. Getnet Chekole (a botanist and associate professor) from Biology Department, College of Natural and Computational Sciences, University of Gondar, with the specimen number GT1, and deposited for future reference. In order to eliminate the dirt and debris on the leaf, the fresh leaf was washed with tap water. Then it was dried at room temperature under shade for two weeks in Department of Pharmacology laboratory room and the dried leaves were crushed into coarse powder.

The article "Antidiarrheal Effect of 80% Methanol Extract and Fractions of Clerodendrum myricoides (Hochst.) Vatke (Lamiaceae) Leaf in Swiss Albino Mice" was published in 2021. Journal: Evid Based Complement Alternat Med.

## 3. Extraction of Plant Material

### 3.1. Preparation of 80% Methanol Extract

The crude methanolic (80%) extract was prepared by cold maceration technique as described by Abdela [31]. One kg of dried and coarsely powdered leaves was weighed by using an electronic balance and soaked in five liters of 80% methanol (MeOH) in Erlenmeyer conical flask for three consecutive days at room temperature. To enhance the extraction process and maximize the yield of extraction, the mixture was occasionally shaken using mini orbital shaker. After three days of maceration, the extract was separated from the marc through a double layer muslin cloth and further filtrated by Whatman No.1 filter paper. In order to exhaustively extract the contents of the leaf, the marc was remacerated twice by adding another fresh solvent in the same way as described above. Once exhaustively extracted, the marc was pressed and filtrated and combined together. Methanol was removed through evaporation by a rotary evaporator which was set at 40°C. The aqueous residue was removed by deep freezing and followed by lyophilization through lyophilizer. Finally, dried 80% MeOH extract was stored in air tight container in deep freezer (−20°C) until it was needed for the required procedure.

### 3.2. Preparation of Fractions

The crude extract was subjected for a successive fractionation using hexane, chloroform, and distilled water as solvents in order of increasing polarity. Seventy gram of extract was suspended in 350 ml of distilled water in a separatory funnel. Then, equal volume of hexane was immersed and the mixture was allowed to form a distinct layer (hexane at the top, the aqueous at the bottom). After 24 hrs, the hexane fraction was removed and the process was repeated twice in the same way with fresh hexane. All the hexane fractions were pooled together and subjected to evaporation via a rotary evaporator which was set at 40°C. Following hexane separation, 350 ml of chloroform was added to the remaining aqueous residue and was allowed to form a separated layer (chloroform at the bottom and aqueous layer at the top). After 24 hrs, the chloroform fraction was partitioned and the process was repeated twice by adding fresh chloroform in the same manner. Chloroform fractions were combined and concentrated using rotary evaporator. The remaining aqueous residue was lyophilized to dryness using lyophilizer. The fractions were labelled and kept in deep freezer with air tight containers until they were used in antidiarrheal test.

The article "Antidiarrheal Effect of 80% Methanol Extract and Fractions of Clerodendrum myricoides (Hochst.) Vatke (Lamiaceae) Leaf in Swiss Albino Mice" was published in 2021. Journal: Evid Based Complement Alternat Med.

### 3.3. Experimental Animals

Either-sex healthy Swiss albino mice that weigh 20–30 g and are 6 to 8 weeks old were used. The mice were handled based on the guidelines for care and use of laboratory animals [32]. The mice were kept and bread in the animal house of University of Gondar, College of Medicine and Health Sciences, School of Pharmacy, Department of Pharmacology. The mice were kept in a standard plastic cage which was bedded with wood chip and had a free access to tap water and a standard pelleted food with a well-controlled temperature and humidity, and 12 hrs dark-light cycle. Mice with age range of 8–12 weeks weighing from 20 to 30 g were selected. Before conducting experimental procedure, all mice were acclimatized for one week to the laboratory conditions.

The care and handling of animals were in accordance with internationally accepted Ethical Guidelines for Laboratory Animals, National Institutes of Health (NIH) Publication No. 86–23, Revised 1985, and the ARRIVE Guidelines.

### 3.4. Animal Grouping and Dosing

For all models, the mice were randomly categorized into five groups with six mice per group. These groups were assigned as negative control and received distilled water for aqueous fractions and 2% Tween 80 in distilled water for the 80% MeOH, chloroform, and hexane fraction. Positive control group received a standard drug loperamide (3 mg/kg orally) for castor oil-induced diarrheal and enteropooling models and atropine (1 mg/kg intraperitoneally) for gastrointestinal motility test model. The test groups received 100, 200, and 400 mg/kg doses based on the acute oral toxicity test from previous study by Reid et al. [29] with limit test dose of 2000 mg/kg. As a result, 10% of the limit dose (200 mg/kg) was selected as middle dose, half of middle dose (100 mg/kg) as lower dose, and twice the middle dose (400 mg/kg) as higher dose. The extracts, distilled water, and loperamide were administered at a volume of 10 ml/kg according to OECD guidelines [33].

### 3.5. Preliminary Phytochemical Screening

The methanolic crude extract was assessed for the presence or absence of flavonoids, tannins, cardiac glycosides, anthraquinones, glycosides, steroids, phenols, terpenoids, alkaloids, and saponins.

## 4. Determination of Antidiarrheal Activity

### 4.1. Castor Oil-Induced Diarrhea

This castor oil-induced diarrhea model was carried out according to the method described by Mekonnen et al. [34]. Thirty Swiss albino mice were fasted for 18 hrs from food with a free access to water and randomly allocated into five groups with six mice per group as described in grouping and dosing section above. After 1 hr administration of the respective doses, each mouse received 0.5 ml of castor oil to induce diarrhea and placed in individual metabolic cage, in which the floor was lined with a white transparent paper for observation of the number and consistency of feces. Then, the paper was changed every hr for 4 hrs duration. During this period of observation, the onset of diarrhea (the time interval in minutes between the administration of castor oil and the appearance of the first diarrheal stool), the number of wet and dry feces, and the weight of fresh feces were recorded.

The article "Antidiarrheal Effect of 80% Methanol Extract and Fractions of Clerodendrum myricoides (Hochst.) Vatke (Lamiaceae) Leaf in Swiss Albino Mice" was published in 2021. Journal: Evid Based Complement Alternat Med.

The total number of wet feces for control group was considered to 100%. Percent inhibition (PI) was calculated as follows:

(1) $$\begin{array}{c} \%\text{ inhibition of diarrhea}=\frac{\text{mean number of wet stools of}\left(\text{negative control group }-\text{ treated group}\right)}{\text{mean number of wet stools of the negative control group}}*100. \end{array}$$

### 4.2. Castor Oil-Induced Enteropooling

This experiment was conducted to evaluate the effect of the plant extract on the inhibition of intraluminal fluid accumulation and done based on the method used by Sisay et al. [35].

Prior to conducting the experiment, the mice were deprived from both food and water for 18 hrs and then received doses (as described in grouping and dosing section). After one hr, the mice received 0.5 ml of castor oil. One hr after administration of castor oil, the mice were sacrificed by cervical dislocation and the abdomen of each mouse was opened and the small intestine (from the pylorus to the caecum) was carefully detached. The small intestine content was weighed and then drained into graduated tube and the volume was measured. Finally, the empty intestine was weighed and the difference between full and empty intestine was calculated.

The percentage of reduction of intestinal secretion (volume and weight) was calculated relative to the negative control based on the following formula:

(2) $$\begin{array}{c} \%\text{ of inhibition by using MVIC}=\frac{\text{MVICC }-\text{ MVICT}}{\text{MVICC}}\times \;100, \end{array}$$

where MVIC is the Mean Volume of Intestinal Content, MVICC is the Mean Volume of Intestinal Content of Control Group, and MVICT is the Mean Volume of Intestinal Content of Test Group.

(3) $$\begin{array}{c} \%\text{ of inhibition by using MWIC}=\frac{\text{MWICC }-\text{ MWICT}}{\text{MWICC}}\times 100, \end{array}$$

where MWIC is the Mean Weight of Intestinal Content, MWICC is the Mean Weight of Intestinal Content of Control Group, and MWICT is the Mean Weight of Intestinal Content of Test Group.

The article "Antidiarrheal Effect of 80% Methanol Extract and Fractions of Clerodendrum myricoides (Hochst.) Vatke (Lamiaceae) Leaf in Swiss Albino Mice" was published in 2021. Journal: Evid Based Complement Alternat Med.

### 4.3. Castor Oil-Induced Gastrointestinal Motility

The method used by Mekonnen et al. [34] was followed to evaluate the effect of 80% MeOH extract and solvent fractions on inhibition of castor oil-induced intestinal motility. The mice were fasted from food for 18 hrs with free access to water and received the respective treatment doses (grouping and dosing). One hr latter, each mouse was given 0.5 ml of castor oil. Then one hr after administration of castor oil, the mice were given a 0.5 ml of charcoal meal (5% activated charcoal in distilled water). The mice were sacrificed by cervical dislocation after half hr of administration of charcoal meal and the small intestine (from the pylorus to caecum) was removed. The distance travelled by the charcoal meal starting from the pylorus toward the caecum and the entire length of the small intestine were measured.

(4) $$\begin{array}{c} \text{Peristalsis index}\left(PI\right)\;=\;\frac{\text{distance travelled by the charcoal meal}}{\text{total length of small intestine}}\times 100,\\ \%\text{ of inhibition }=\;\frac{\text{PI of negative control }-\text{ PI of drug or extract treated}}{\text{PI of negative control}}\times 100. \end{array}$$

### 4.4. *In Vivo* Antidiarrheal Index (ADI)

The *in vivo* antidiarrheal index (ADI) for the 80% MeOH extract, solvent fractions, and standard drug was calculated by combining three parameters which were taken from the aforementioned models and based on the following formula [36]:

(5) $$\begin{array}{c} \text{ADI in vivo}=\;\sqrt[{3}]{\text{Dfreq}*\text{Gmeq}*\text{Pfreq}}, \end{array}$$

where Dfreq is the delay in the onset of diarrhea compared to the negative control (as % of control), Gmeq is reduction in distance moved by the charcoal meal compared to negative control (as % of control), and Pfreq is the purging frequency or the reduction in the number of wet feces compared to the negative control (as % of control).

Each parameter was calculated based on the following formula:

(6) $$\begin{array}{c} \text{Dfreq}=\frac{\text{mean onset of diarrhea}\left(\text{in treated group}-\text{in the negative control group}\right)}{\text{mean onset of diarrhea in the negative control group}}\times 100,\\ \text{Gmeq }=\;\frac{\text{distance travelled by the charcoal meal in the}\left(\text{control }-\text{test}\right)\text{group}}{\text{distance travelled by the charcoal meal in the control group}}\times 100,\\ \text{Pfreq}=\frac{\text{mean number of wet feces of}\left(\text{control}-\text{treated}\right)\text{group}}{\text{mean number of wet feces of the control group}}\times 100. \end{array}$$

The article "Antidiarrheal Effect of 80% Methanol Extract and Fractions of Clerodendrum myricoides (Hochst.) Vatke (Lamiaceae) Leaf in Swiss Albino Mice" was published in 2021. Journal: Evid Based Complement Alternat Med.

### 4.5. Statistical Analysis

The results of the experiments were managed and analyzed by using Statistical Package for Social Sciences (SPSS) software version 23. The outcomes from the SPSS analysis were presented as mean ± standard error of mean (SEM). The statistically significant difference between groups and within groups was carried out via One-Way Analysis of Variance (ANOVA) followed by Tukey's post hoc multiple comparison test. The result was considered statically significant when the *P* value was less than 0.05 at 95% confidence interval.

## 5. Results

### 5.1. Preliminary Phytochemical Screening

The result from phytochemical analysis of the of the crude extract has shown the presence tannins, flavonoids, alkaloids, saponins, terpenoids, steroids, phenols, and anthraquinones while glycosides were absent.

### 5.2. Effects on Castor Oil-Induced Diarrhea

In the course of 4 hrs observation after castor oil was administered, the antidiarrheal effect of the 80% MeOH extract and solvent fractions of the leaf of *C. myricoides* on castor oil-induced diarrhea are presented in Table 1. Compared to negative control, 80% MeOH extract of the leaf of *C. myricoides* significantly prolonged the onset of diarrhea at 200 (*P* < 0.01) and 400 mg/kg doses (*P* < 0.001) and reduced the number of wet feces, total number of feces, and weight of fresh feces at all tested doses. The percentage of diarrhea inhibition by the extract was 47.33% (*P* < 0.05), 54.53% (*P* < 0.001), and 69.14% (*P* < 0.001) at 100, 200, and 400 mg/kg, respectively.

Both chloroform and aqueous fractions significantly prolonged the onset of diarrhea at 200 mg/kg and 400 mg/kg compared to the negative control. All tested doses of chloroform fraction produce a significant reduction on the number of wet feces, total feces, and the weight of fresh feces. On the contrary, the hexane fraction showed a significant effect at all parameters only at 400 mg/kg dose as compared with the negative control with 45.47% (*P* < 0.05) of diarrhea inhibition. The percentage of diarrhea inhibition by chloroform fraction at 100, 200, and 400 mg/kg was 43.62% (*P* < 0.05), 50.92% (*P* < 0.01), and 65.43% (*P* < 0.001), respectively. The percentage of diarrhea inhibition by 200 and 400 mg/kg dose of the aqueous fraction was 52.49% (*P* < 0.01) and 62.84% (*P* < 0.001).

### 5.3. Effects on Castor Oil-Induced Enteropooling

In the evaluation of castor oil-induced fluid accumulation (enteropooling) model which is presented in Table 2, 80% MeOH extract and chloroform fraction of the leaf of *C. myricoides* revealed a significant reduction in both volume and weight of intestine contents at all tested doses when compared to the negative control group.

The article "Antidiarrheal Effect of 80% Methanol Extract and Fractions of Clerodendrum myricoides (Hochst.) Vatke (Lamiaceae) Leaf in Swiss Albino Mice" was published in 2021. Journal: Evid Based Complement Alternat Med.

The percentage of volume reduction by 80% MeOH extract was found to be 33.33%, (*P* < 0.01), 44.00% (*P* < 0.001), and 53.33% (*P* < 0.001), and the weight reduction was 35.71% (*P* < 0.01), 45.24% (*P* < 0.001), and 55.95% (*P* < 0.001) at 100, 200, and 400 mg/kg doses, respectively. The percentage of volume reduction by chloroform fraction at 100, 200, and 400 mg/kg was 30.67% (*P* < 0.05), 40.00% (*P* < 0.01), and 54.69% (*P* < 0.001), respectively. At these respective doses, the percentage of weight reduction was 34.52% (*P* < 0.05), 44.05% (*P* < 0.001), and 53.57% (*P* < 0.001).

The aqueous fraction at 200 and 400 mg/kg demonstrated a significant reduction in both volume and weight of the intestinal contents compared to the negative group. The percentage of reduction in volume was 38.16% (*P* < 0.01) and 44.74% (*P* < 0.001), and in weight it was 40.23% (*P* < 0.01) and 49.43% (*P* < 0.001) at 200 and 400 mg/kg doses, respectively. On the other hand, the hexane fraction showed a significant reduction in volume (32.00%) and weight (32.14%) of intestinal contents only at the 400 mg/kg (*P* < 0.05) (Table 2).

### 5.4. Effects on Castor Oil-Induced Gastrointestinal Motility

When compared to the negative control group, the crude extract significantly reduced the distance travelled by charcoal meal at 100, 200, and 400 mg/kg with the percentage of inhibition 42.57% (*P* < 0.01), 55.29% (*P* < 0.001), and 63.55% (*P* < 0.001), respectively. The inhibition of charcoal meal transit by the 400 mg/kg dose was closely related with the standard drug atropine sulfate, being 67.27%.

The percentage of reduction in the transit of charcoal meal by chloroform fraction was 38.88% (*P* < 0.01), 53.24% (*P* < 0.001), and 59.88% (*P* < 0.001) at 100, 200, and 400 mg/kg, while the percentage reduction of gastrointestinal transit for aqueous fraction at the 200 mg/kg and 400 mg/kg was 45.13% (*P* < 0.01) and 50.08% (*P* < 0.001). Hexane fraction produced a significant decrease in the movement of the charcoal meal along the lumen of intestine only at the dose of 400 mg/kg (32.97%, *P* < 0.05) as compared to the control group (Table 3).

### 5.5. *In Vivo* Antidiarrheal Index

The ADI is a measure of the combined effects of different diarrhea evaluation parameters to determine the relative antidiarrheal activity of the crude extract and solvent fractions. The highest ADI was observed at the maximum dose of 80% MeOH crude extract (82.59%), which was nearly similar to the standard drug (Table 4). Furthermore, the highest ADI was observed at the maximum dose of each fraction. Among the solvent fractions, the chloroform fraction showed the highest ADI value, which was 78.51%, and the lowest ADI was exhibited by hexane fraction.

The article "Antidiarrheal Effect of 80% Methanol Extract and Fractions of Clerodendrum myricoides (Hochst.) Vatke (Lamiaceae) Leaf in Swiss Albino Mice" was published in 2021. Journal: Evid Based Complement Alternat Med.

## 6. Discussion

The leaf of *C. myricoides* is a commonly utilized plant for the treatment of diarrhea in different parts of the Ethiopia without scientific proof for its efficacy and safety. Basically in the traditional practice, the leaf of *C. myricoides* is taken by using water as vehicle; however, in this study 80% methanol was used. Methanol is highly soluble in water. Methanol has high extraction yield and greater potential in extracting wide range of plant phytochemical constituents [37]. Furthermore, methanol is unsuitable for the proliferation of pathogenic microorganisms. Additionally, hydromethanolic extract can be easily suspended in distilled water during fractionation [38]. Therefore, 80% MeOH was used as a solvent in this study for the initial extraction of the leaf of *C. myricoides*.

The finding in this research is comparable to the results reported from the aqueous and chloroform fraction of the root of *C. abyssinica* [39]. The antidiarrheal effect of 80% MeOH extract and solvent fraction was dose dependent. Moreover, the highest percent of antidiarrheal activity was observed at 400 mg/kg dose of extracts, indicating the highest doses of the extracts can better accumulate antidiarrheal bioactive compounds both in quantity and in quality.

The antidiarrheal activity of the medicinal plants might be due to the presence of secondary metabolites such as flavonoids, alkaloids, tannins, saponins, phenols, terpenoids, steroids [40, 41]. In this study, the phytochemical screening test of the 80% MeOH extract revealed the presence of alkaloids, flavonoids, tannins, saponins, phenols, steroids, terpenoids, and anthraquinones. These phytochemicals exert antidiarrheal activity through different mechanisms. Tannins and flavonoids increased colonic water and electrolyte reabsorption. Flavonoids and terpenoids inhibited the release of autacoids and prostaglandins. Phenols inhibit intestinal secretion and motility [42]. Additionally, an earlier *in vitro* study revealed that methanolic extract of leaf of *C. myricoides* has marked inhibition of lipopolysaccharide stimulated nitric oxide synthesis [28]. Diarrhea due to castor oil has been enhanced by nitric oxide through facilitation of intestinal secretion and motility [43]. Hence, the extract's ability to inhibit nitric oxide pathway might be one of the antidiarrheal mechanisms.

Castor oil also causes diarrhea by increasing oxidative stress on the intestinal epithelium which in turn alters the movement of electrolytes and water through the intestinal mucosa [44]. It is proved that the leaf of *C. myricoides* has antioxidant properties which may account for another antidiarrheal mechanism [18]. From the previous *in vitro* study, the extracts of the leaf of *C. myricoides* demonstrated inhibition of cyclooxygenase, an enzyme responsible for the synthesis of prostaglandins [27]. Prostaglandin stimulates the secretion of intestinal fluid and electrolytes and decreases absorption of glucose [45, 46], which might be another antidiarrheal mechanism of the plant. Tannins are known to have antidiarrheal activity by denaturing proteins through the formation of protein tannate in intestinal mucosa making it more resistant to chemical alteration thereby reducing secretion [47]. Flavonoids and steroids were identified as inhibitor of cyclooxygenase and lipoxygenase, in turn inhibiting prostaglandin induced fluid secretion [48]. Steroids are also known for their enhancement of water and sodium absorption [49].

The article "Antidiarrheal Effect of 80% Methanol Extract and Fractions of Clerodendrum myricoides (Hochst.) Vatke (Lamiaceae) Leaf in Swiss Albino Mice" was published in 2021. Journal: Evid Based Complement Alternat Med.

The extract of the plant has shown antimotility activity in dose dependent manner. Decreased intestinal motility increases the contact time of intestinal contents for absorbing surfaces in the lumen, which can increase water and electrolyte absorption. The antimotility action of both 80% MeOH extract and the solvent fractions might be attributed to the presence of phytochemicals. Alkaloids isolated from the plant showed antispasmodic activity on isolated guinea pig ileum [50]. Flavonoids produced antimotility activity through *α*_2_-adrenergic receptors stimulation and the inward calcium current hindering [51]. Tannins have spasmolytic and smooth muscle relaxant effect by decreasing the intracellular Ca^2+^ inward current and through facilitating calcium pumping system [47]. *α*-terpineol, which was identified in this plant, also demonstrated antimotility activity in bethanechol induced intestinal contraction [52].

Antidiarrheal index denotes the combined effects of three diarrheal parameters such as purging frequency in number of wet feces and delay in onset of diarrheal stool and intestinal motility. The higher the ADI value, the greater the effectiveness of the extract in the treatment of diarrhea [25]. The highest ADI value was produced by the 80% MeOH extract at its high dose which is directly related to its efficacy in treating diarrhea.

## 7. Conclusion

This study has shown that the leaves of *C. myricoides* have constituents responsible for significant antidiarrheal activity which supports the claimed traditional medical practice.

## Figures and Tables

**Table 1:** The effects of 80% methanol extract and solvent fractions of the leaf of *C. myricoides* on the castor oil-induced diarrheal model in mice.

Dose (mg/kg)	Onset of diarrhea	Number of wet feces	Total number of feces	Weight of fresh feces	% diarrhea inhibition
Control	53.43 ± 5.79	9.17 ± 1.17	11.50 ± 1.05	0.38 ± 0.04	—
MeOH 100	73.60 ± 6.97^c2b3^	4.83 ± 0.31^a1b3c3^	6.17 ± 0.31^a1b2c3^	0.22 ± 0.04^a2c1^	47.33
MeOH 200	98.27 ± 3.79^a2b2c2^	4.17 ± 0.62^a3b2c2^	5.33 ± 0.56^a3^	0.16 ± 0.02^a3^	54.53
MeOH 400	121.93 ± 2.17^a3^	2.83 ± 0.31^a3^	4.67 ± 0.42^a3^	0.13 ± 0.01^a3^	69.14
Lop 3	134.77 ± 3.80^a3^	2.50 ± 0.22^a3^	4.00 ± 0.40^a3^	0.10 ± 0.02^a3^	72.74
HF 100	57.43 ± 5.31^b2c3^	7.83 ± 0.48^b2c3^	10.67 ± 1.02^b3b3^	0.33 ± 0.02^b3c3^	14.61
HF 200	63.27 ± 0.61^b2c3^	7.17 ± 0.60^b3c3^	9.83 ± 0.75^b3c3^	0.29 ± 0.02^b2c3^	21.81
HF 400	86.10 ± 7.9^a2b2c3^	5.00 ± 0.32^a1b2c2^	7.33 ± 0.71^a1b2c2^	0.23 ± 0.02^a1b2c2^	45.47
CF 100	67.77 ± 5.32^b2c2^	5.17 ± 0.31^a1b2c2^	7.83 ± 0.33^a1b2c3^	0.25 ± 0.04^a1c1^	43.62
CF 200	94.60 ± 5.91^a2b2^	4.50 ± 0.56^a2^	6.33 ± 0.48^a1^	0.19 ± 0.02^a3^	50.92
CF 400	119.43 ± 4.32^a3^	3.17 ± 0.31^a3^	4.50 ± 0.72^a3^	0.15 ± 0.01^a3^	65.43

Control	47.64 ± 4.66	9.83 ± 0.31	11.83 ± 0.33	0.37 ± 0.05	—
AF 100	59.48 ± 2.89^b2c3^	6.83 ± 0.48^b2c3^	8.67 ± 0.33^b2c3^	0.28 ± 0.03^b2c2^	30.52
AF 200	82.48 ± 4.98^a2b2c2^	4.67 ± 0.49^a2^	6.50 ± 0.67^a2c3^	0.22 ± 0.02^a2^	52.49
AF 400	107.81 ± 4.37^a3^	3.67 ± 0.33^a3^	5.00 ± 0.37^a3^	0.18 ± 0.02^a3^	62.67
Lop 3	128.17 ± 3.80^a3^	2.67 ± 0.22^a3^	4.00 ± 0.40^a3^	0.12 ± 0.02^a3^	72.84

Values are expressed as mean ± standard error of mean (*n* = 6), ^a^compared to the negative control, ^b^compared to the 400 mg/kg MeOH extract, and ^c^compared to the positive control. MeOH: 80% methanol extract; Lop 3: 3 mg/kg loperamide; CF: chloroform fraction; HF: hexane fraction; AF: aqueous fraction. Controls were given 10 ml/kg distilled water (for aqueous fraction) and 10 mk/kg of 2% Tween 80 (for chloroform fraction, hexane fraction, and crude extract). ^1^*P* < 0.05, ^2^*P* < 0.01, and ^3^*P* < 0.001.

The article "Antidiarrheal Effect of 80% Methanol Extract and Fractions of Clerodendrum myricoides (Hochst.) Vatke (Lamiaceae) Leaf in Swiss Albino Mice" was published in 2021. Journal: Evid Based Complement Alternat Med.

**Table 2:** The effects of 80% methanol extract and solvent fractions of the leaf of *C. myricoides* on the castor oil-induced enteropooling model in mice.

Dose (mg/kg)	VSIC (ml)	% of volume inhibition	WSIC (g)	% of weight inhibition
Control	0.75 ± 0.03	—	0.84 ± 0.03	—
MeOH 100	0.50 ± 0.02^a2b1c3^	33.33	0.54 ± 0.03^a2b1c3^	35.71
MeOH 200	0.42 ± 0.03^a3^	44.00	0.46 ± 0.05^a3^	45.24
MeOH 400	0.35 ± 0.03^a3^	53.33	0.37 ± 0.03^a3^	55.95
Lop 3	0.30 ± 0.03^a3^	60.00	0.33 ± 0.03^a3^	60.71
HF 100	0.68 ± 0.03^b3c3^	9.33	0.72 ± 0.03^b3c3^	14.29
HF 200	0.60 ± 0.05^b2c3^	20.00	0.68 ± 0.05^b2c3^	19.05
HF 400	0.51 ± 0.03^a1b2c3^	32.00	0.57 ± 0.04^a1b1c2^	32.14
CF 100	0.52 ± 0.07^a1b1c3^	30.67	0.55 ± 0.05^a1b3c1^	34.52
CF 200	0.45 ± 0.04^a3^	40.00	0.47 ± 0.03^a3^	44.05
CF 400	0.34 ± 0.02^a3^	54.69	0.39 ± 0.06^a3^	53.57

Control	0.76 ± 0.02	—	0 .87 ± .04	—
AF 100	0.55 ± 0.03^b2c3^	27.63	0.64 ± 0.03^b3c3^	26.44
AF 200	0.47 ± 0.02^a2b2^	38.16	0.52 ± 0.03^a2b1c1^	40.23
AF 400	0.42 ± 0.04^a3^	44.74	0 .44 ± 0.01^a3^	49.43
Lop 3	0.33 ± 0.03^a3^	56.58	0.35 ± 0.02^a3^	59.77

Values are expressed as mean ± standard error of mean (*n* = 6), ^a^compared with the negative control, ^b^compared with the 400 mg/kg MeOH extract, and ^c^compared with the positive control. VSIC (ml): volume of the small intestinal content; WSIC (g): weight of the small intestinal content; MeOH: 80% methanol extract; Lop: loperamide; CF: chloroform fraction; HF: hexane fraction; AF: aqueous fraction. Controls were given 10 ml/kg 2% Tween 80 (for 80% MeOH extract, chloroform, and hexane fractions) and 10 ml/kg distilled water (for aqueous fraction). ^1^*P* < 0.05, ^2^*P* < 0.01, and ^3^*P* < 0.001.

**Table 3:** The effects of 80% MeOH extract and solvent fractions of the leaf of *C. myricoid*es on castor oil-induced gastrointestinal motility in mice.

Treatment (mg/kg)	LSI (cm)	DTCM (cm)	PI	% inhibition
Control	52.54 ± 1.54	36.69 ± 2.39	69.83 ± 4.24	—
MeOH 100	56.93 ± 1.34	22.83 ± 1.78^a2b1c3^	40.10 ± 3.21^a2b1c1^	42.57
MeOH 200	55.50 ± 1.91	17.33 ± 3.57^a3^	31.23 ± 2.29^a3^	55.29
MeOH 400	54.33 ± 1.23	13.83 ± 0.91^a3^	25.46 ± 1.83^a3^	63.55
Atr 1	53.25 ± 0.96	12.17 ± 0.91^a3^	22.85 ± 1.76^a3^	67.27
HF 100	56.75 ± 1.14	33.00 ± 2.59^b3c^	58.15 ± 3.90^b3c3^	16.73
HF 200	58.17 ± 1.85	30.58 ± 2.89^b3c3^	52.57 ± 5.89^b3c3^	24.72
HF 400	56.08 ± 0.93	26.25 ± 2.29^a1b2c3^	46.81 ± 3.77^a1b2c2^	32.97
CF 100	54.17 ± 2.41	23.12 ± 1.74^a2b1c3^	42.68 ± 3.22^a2b1c3^	38.88
CF 200	57.17 ± 1.62	18.67 ± 1.26^a3^	32.66 ± 2.68^a3^	53.24
CF 400	53.25 ± 0.91	14.92 ± 1.51^a3^	28.02 ± 2.96^a3^	59.88

Control^2^	55.58 ± 0.76	40.08 ± 1.58	72.11 ± 3.67	—
AF 100	55.24 ± 1.82	28.8 ± 1.45^b2c3^	52.14 ± 1.55^b2c3^	27.70
AF 200	53.50 ± 0.96	21.17 ± 0.87^a2c2^	39.57 ± 2.23^a2c2^	45.13
AF 400	55.50 ± 1.55	19.98 ± 1.37^a3^	36.00 ± 1.92^a3^	50.08
Atr 1	54.83 ± 1.19	13.90 ± 0.99^a3^	25.35 ± 2.03^a3^	64.84

Values are expressed as mean ± standard error of mean (*n* = 6), ^a^compared to the negative control, ^b^compared to the 400 mg/kg MeOH extract, and ^c^compared to the positive control. LSI (cm): length of the small intestine; DTCM (cm): distance travelled by charcoal meal; PI: peristalsis index; MeOH: 80% methanol extract; Atr: atropine; HF: hexane fraction; CF: chloroform fraction; AF: aqueous fraction. Controls were given 10 ml/kg distilled water (for aqueous fraction) and 10 ml/kg 2% Tween 80 (for 80% MeOH extract, chloroform, and hexane fractions). ^1^*P* < 0.05, ^2^*P* < 0.01, and ^3^*P* < 0.001.

The article "Antidiarrheal Effect of 80% Methanol Extract and Fractions of Clerodendrum myricoides (Hochst.) Vatke (Lamiaceae) Leaf in Swiss Albino Mice" was published in 2021. Journal: Evid Based Complement Alternat Med.

**Table 4:** *In vivo* antidiarrheal index of 80% MeOH and solvent fractions of *C. myricoides* leaf.

Treatment (mg/kg)	Delay in diarrhea (minute)	Gut meal travel distance (Gmeq) (%)	Purging frequency (Pfreq) (%)	Antidiarrheal index (ADI)
MeOH 100	37.75	42.57	47.33	42.37
MeOH 200	83.92	55.29	54.53	63.25
MeOH 400	128.21	63.55	69.14	82.59
PC	152.24	67.27	72.74	90.65
HF 100	7.49	16.73	14.61	12.23
HF 200	18.42	24.72	21.81	21.23
HF 400	61.15	32.97	45.47	45.09
CF 100	26.84	38.88	43.62	35.71
CF 200	77.05	53.24	50.92	59.33
CF 400	123.53	59.88	65.43	78.51
AF 100	24.85	32.26	30.52	29.03
AF 200	73.13	42.16	52.49	54.50
AF 400	126.30	58.00	62.67	77.14
PC	169.04	64.82	72.84	92.7 6

Values are expressed as mean ± standard error of mean (*n* = 6). MeOH: 80% methanol extract; HF: hexane fraction; CF: chloroform fraction; AF: aqueous fraction; PC: positive control (atropine 1 mg/kg and loperamide 3 mg/kg); Dfreq: delay in diarrhea onset (in % of control). Gmeq is the intestinal meal travel reduction (in % of control). Pfreq is the purging frequency as the number of wet feces' reduction (in % of control).

## Data Availability

The datasets used and/or analyzed during the study are available from the corresponding author upon reasonable request.
